The article "Analysis Model of the Influence of Self-Efficacy on Professional Toughness of Preschool Teachers under the Condition of Ensuring Children's Mental Health and Healthy Family Environment" was retracted in 2023. Reasons: unreliable results or conclusions; concerns about the data; concerns about the results or conclusions; concerns about the peer review.

# Analysis Model of the Influence of Self-Efficacy on Professional Toughness of Preschool Teachers under the Condition of Ensuring Children's Mental Health and Healthy Family Environment

**DOI:** 10.1155/2022/3737690

**Published:** 2022-09-27

**Authors:** Yanfang Zhou, Yuping Wu, Xiaojie Deng, Sihui Wang, Leishan Shi

**Affiliations:** ^1^Lishui University, Lishui 323000, China; ^2^Zhejiang Sci-Tech University, Hangzhou 310018, China; ^3^Ningbo University, Ningbo 315211, China

## Abstract

Preschool teachers' professional toughness (PT) has received a lot of attention recently, and this research is one of the main areas of study for their ability to manage stress and develop normally. Based on how well a person thinks of his own abilities, SE (self-efficacy) is formed. 300 kindergarten teachers from 10 metropolitan kindergartens were chosen as research samples in order to examine the relationship between the SE of kindergarten teachers and their PT, as well as the mediating effects of professional identity and work passion. A paradigm for measuring teacher performance based on the BPNN (BP neural network) is proposed, and several data processing techniques are developed. The study's findings indicate that teachers' WE (work enthusiasm) fills a limited intermediary role between PT and SE; the intermediary effect value is 0.041 and accounts for 15.7% of the overall effect (0.6559). The conclusion is that in order to help new instructors cope with their negative feelings, it is important to engage in a variety of leisure activities.

## 1. Introduction

Helping students know themselves, accept themselves, and develop their potential is the main goal of school psychological counseling. Whether students can succeed in study, life, and social interaction is closely related to their positive self-belief. New kindergarten teachers generally have some problems, such as double marginalization, lack of competitiveness in the salary level, neglect of education rights, low professional reputation, and high turnover rate and tendency. The teachers' group needs attention. However, the high mobility and instability of preschool teachers is a long-standing problem, and the frequent turnover of teachers will not only harm the learning and development of preschool children [1]. The level of preschool teachers' PT (professional toughness) affects not only the quality of life of preschool teachers but also their recognition and satisfaction with preschool teachers' profession, as well as their physical and mental health. Therefore, it is very urgent and necessary to study the PT of preschool teachers.

In addition to completing the most basic education work, teachers should coordinate the relationships among kindergartens, families, society, and children. Preschool PT refers to the ability of preschool teachers to overcome difficulties, cope with pressure, and rejuvenate themselves by adopting various coping styles when they encounter various difficulties in their work. WE (work enthusiasm) stands for a positive, full-hearted, and heart-driven working state, and individuals with high WE will spontaneously and actively devote themselves to work. I hope that the individual organization will be energetic and dedicated to the work and make due contributions to the work [2]. A strong psychological resilience can help kindergarten instructors overcome obstacles in their work and persevere under pressure. This essay shows the significance of psychological resilience in the process of teachers' professional growth by investigating the circumstances and traits of psychological resilience in preschool teachers from a scientific perspective. Burnout at work is a psychological barrier to teachers' progress that impacts their sense of accomplishment, professional development, relationships with pupils, and physical and mental health. It also has a negative psychological impact on their sense of self-growth. There is a relationship between these three elements and how they affect teachers' work attitudes, work performance, and physical and mental health [3].

SE (self-efficacy) is relatively stable, and its early situation affects its later development. Therefore, helping children to form a higher level of SE is of positive significance to their physical and mental development. Fundamentally speaking, professional adaptation and PI (professional identity) are intertwined and influence each other, both of which are individuals' psychological cognition and psychological state of professional activities. Teachers do not get enough support in the process of SE construction. When they experience negative events, they will gradually lose their satisfaction and commitment to their work. Starting from the individual factors that affect teachers' work behavior, this study selects PI variables in cognitive factors and SE variables in emotional factors and tries to reveal the influence of SE on kindergarten teachers' PT and the relationship between PI, WE, and kindergarten teachers' work behavior. On the other hand, it also provides theoretical support for the research of kindergarten teachers' PI and SE development, which has strong theoretical significance.

Research innovation includes the following:

1. This study introduced SE into the field of education, discussed the relationship between kindergarten teachers' work behavior and PI and SE, further analyzed the intermediary role of SE between them, profoundly revealed the occurrence and development mechanism of kindergarten teachers' work behavior, and further supplemented the research on influencing factors of kindergarten teachers' work behavior
2. According to the actual situation, classify the outliers in the teacher assessment system, study the outlier diagnosis algorithm suitable for the teacher assessment system, and make effective corrections for different types of outliers so as to minimize the impact of outliers on the final evaluation grade of teachers

The following describes the general structure of this article. The background work for the research is presented in Section 1.  Section 2 mostly introduces the current context of this investigation. The realization design of the research model is presented in Section 3. The effectiveness of the model under study in this research is confirmed in Section 4. The conclusion is found in Section 5.

## 2. Related Work

### 2.1. The Related Research of SE

Tsai believes that the size of the school, the state of the school's organizational atmosphere, students' performance, and teachers' own cognitive processing have an impact on SE [4]. Lent et al. found that SE played a moderating role between job stress and job burnout of primary and secondary school teachers [5]. Nikolaus et al. investigated 1059 middle school teachers with an SE questionnaire, school organizational innovation questionnaire, and teaching innovation questionnaire and found that SE of middle school teachers was significantly related to the school organizational innovation atmosphere [6]. Roberts et al. investigated 135 preschool teachers in Zhanjiang by using the Teacher SE Scale to explore the influence of related factors on preschool teachers' SE. The results show that SE has achieved significant differences in marital status [7].

### 2.2. The Related Research of PT

Constantino et al. believe that PT is the individual competitiveness and adaptability of preschool teachers in the ever-changing preschool teaching environment [8]. Ling et al. summarized the influencing factors of teachers' primitiveness, including internal factors and external factors. Internal factors include positive personality traits, a sense of professional accomplishment, and PI, while external factors include leadership support, teaching policies and incentives, and colleagues' relationships [9]. Visser et al. concluded that personality will affect teachers' psychological recovery, and a cheerful personality is conducive to improving psychological recovery [10]. Understanding the objective occupation is conducive to the promotion of psychological resilience. Getting to know children better is conducive to the improvement of psychological resilience. The research of Urbániková and Volek shows that the professional toughness of township PE teachers is significantly higher than that of urban PE teachers, and the self-improvement ability of urban PE teachers is significantly higher than that of township PE teachers [11].

### 2.3. Research on the Relationship between SE and PT

Sundberg et al. think that there is a significant positive correlation between self-efficacy and toughness. The higher your self-efficacy is, the more you dare to face difficulties, and you will not flinch easily, and the higher your toughness level will be [12]. According to Nowicka's research, the SE of English teachers in independent colleges has a certain influence on resilience, and then a series of suggestions are put forward to enhance SE and develop resilience through the attention of the management level [13]. Walker and Rossi found that there was a significant difference in the sense of efficacy between kindergarten teachers in the high-toughness group and those in the low-toughness group and then put forward a series of targeted educational suggestions [14].

### 2.4. Literature Review of PI

PI stands for the extent of a person's occupation's acceptability and acknowledgment. Three areas dominate the meaning of PI: attitude intention, characteristic intention, and identification intention. The characteristics of centrality, value, interpersonal unity, and self-presentation should be included in a teacher's performance indicators, according to Ings. Sex draws attention to its inner sense perception [15]; Hamming investigated the dimensions of teachers' professional identities (PI) and uncovered nine of them, including professional ability, professional significance, characteristic cognition, leadership identity, colleague identity, student identity, professional reward identity, work situation identity, and affiliation with educational institutions like schools [16]. Steinberg and Kraft used the stratified sampling method to investigate the relationship between kindergarten teachers' mental health and professional ethics. They also built an intermediary adjustment model and discovered that mental health can affect professional ethics through the transmission of PI [17].

### 2.5. Literature Review of WE

WE reflects that individuals deeply combine, embed, and integrate the norms, responsibilities, and contents required by their job roles and use physiological, cognitive, and psychological energy to perform their job roles, highlighting their sense of identity with their job roles. It can be seen that WE can be a positive output of results, which not only promotes their career development but also helps to improve organizational efficiency.

Doan et al. describe WE as the embedding degree of an individual's job role, which reflects an individual's recognition and commitment to work, while job burnout is the negative embodiment of WE [18]. Li thinks WE is a dual state of work-related factors, cognitive and emotional, and proposes that WE has three dimensions, namely, vitality, dedication, and concentration [19]. Anderson and Collis collected relevant data of primary school teachers for investigation and found that teachers' WE consists of three dimensions by factor analysis, which are work importance, work focus, and work pleasure [20, 21].

## 3. Methodology

### 3.1. Research Model Design

In the face of pressure and challenges, PT is the necessary guarantee for preschool teachers to be competent, and it is also an important condition for preschool education. Children spend their whole day in kindergarten and have a lot of communication with their peers. However, teachers' words also play a great role. In front of teachers, children always want to do their best and be praised. However, some children's personal ability is weak. For these children, when they have finished their task, if teachers do not give timely praise and compare them with children with better abilities, then their SE will be difficult to improve or even lower.

PI includes six dimensions: professional knowledge, professional expectations, professional will, professional skills, professional emotions, and professional values. Satisfaction is a relative concept, a concept corresponding to individual expectations and experiences, and a state at the same time. This word originated from the field of economics at first, and it is a kind of pleasure after customers' expectations or needs are realized or satisfied. Subjectivity means that teachers' job satisfaction has a certain subjective color. Level means that the satisfaction of teachers will vary with the teachers' individuality and their age and career stage, and their subjective feelings will be different, and they will change with the changes of the external environment and the development of the industry prospect, exceeding the excessive requirements of personal energy and resources, resulting in mental, emotional, and behavioral exhaustion.

PT has the following characteristics. First, individuals encounter setbacks and difficulties and bear psychological trauma or pressure. Second, individuals can use their internal protective resources, including abilities, cognitive and psychological characteristics, and external support, including family support, social support, and kindergarten support. PT is an individual's ability to bounce back from a career dilemma, especially the ability to persist in a bad career environment. This study holds that PT is an individual's positive psychological characteristic and behavior tendency that can overcome difficulties and adapt to the environment through internal protective factors such as optimism, self-confidence, courage, and positive explanation and external supportive factors after encountering difficulties and setbacks in work and bearing certain pressure.

PI is a one-dimensional structure. A six-item scale of PI has been developed, which is suitable for PI evaluation in different industries. The scale has good reliability and validity and has been widely used in empirical research. Kindergarten teachers often need more superior and ideal working environments and conditions to realize their PI. Once kindergartens provide them with external incentives that meet the inherent needs of preschool teachers, they will be stimulated to have a strong PI. PI is usually related to organizational characteristics and is generally affected by organizational competition and organizational image and reputation. The two are not mutually exclusive but depend on each other and work together. Related research shows that teachers' double identity can effectively explain their attitudes and behaviors. Based on this, the author speculates that compared with other double identity combinations, the double identity combination of kindergarten teachers with high PI has the most significant positive impact on their WE.

This study tries to find out the current situation of preschool teachers' PI sense, SE, and WE through the investigation of preschool teachers' groups, explore the relationship among them, discuss the influencing factors of preschool teachers' PI, SE, and WE, find out the causes of influencing preschool teachers' WE, and then put forward corresponding educational suggestions.

Therefore, the following research hypotheses are put forward.

**Hypothesis 1 .**

Preschool teachers' PI, WE, and SE are different in age, teaching years, monthly salary, kindergarten location, educational background, labor relations, and marital status.

**Hypothesis 2 .**

Four dimensions of kindergarten teachers' PI professional values, role values, professional sense of belonging, and professional behavior tendency can positively influence WE.

**Hypothesis 3 .**

Both teachers' PI and job satisfaction can predict job burnout, and they are negative predictors.

**Hypothesis 4 .**

SE of preschool teachers plays an intermediary role in the influence of social support on PT.

Based on the correlation among the new kindergarten teachers' professional adaptation, PI and its internal factors, and professional development support and its internal factors, this study assumes that, with professional adaptation as an independent variable, PI and its three internal factors as dependent variables, and professional development support and its four internal factors as intermediary variables, a hypothetical model of the intermediary effect among them is constructed.  Figure 1 shows the research model design.

### 3.2. Diagnosis and Correction of Outliers in Teachers' Peer Evaluation Data

To maintain preschoolers' safety in the kindergarten, teachers should pay attention to both their physical and mental health in addition to their mental education and meeting their growth demands. As a result, the work behavior of instructors comprises “WE,” which is good for education, as well as instructional behavior and conservation behavior. Additionally, encourage children to behave well. Teachers' active WE can coordinate different educational influences and give kids a positive home environment. As a result, encouraging preschoolers' harmonic development depends greatly on the work behavior of excellent teachers. Kindergarten teachers are experts with advanced educational concepts, professional knowledge, and educational skills. They can affect preschoolers' education by fusing academic ideas with social expectations, work demands, and many other variables. Therefore, in-depth and meticulous research must be done on preschool teachers' work behavior in order to provide an effective theoretical foundation for improving the benign development of preschool teachers' work behavior in China and to promote the healthy growth of preschool children at this stage.

Carrying out teacher performance evaluation is the need of deepening the reform of the school internal management system and strengthening management efficiency. Deepening the school internal management system involves a wide range of heavy tasks, but the core is the management of teachers. The process of evaluating teachers' performance is the process of checking, guiding, assessing, and supervising each teacher's work, and it is a scientific and orderly management process. Therefore, in order to improve teachers' teaching and scientific research level, enhance the management level of school education and teaching, further deepen the reform of the education system, and improve the competitiveness of schools, every school urgently needs to establish a teacher performance evaluation system that meets its own needs.

The major method used by schools to accomplish their educational objectives is classroom instruction. In order to fully and completely comprehend the state of school teaching, as well as to enhance teaching quality, school administrators and managers will benefit from evaluating the effectiveness of teachers' classroom instruction. Some students fill out their data and submit them as a result of their mistakes throughout the operation process, while others enter incorrect information, which can result in unclean or lost data. Therefore, the primary technique for resolving the aforementioned issues is the introduction of scientific calculating methods. Paper evaluation forms are typically used in traditional teaching quality evaluations, which not only wastes resources but also significantly lowers the effectiveness of the evaluation. The networking of the evaluation process will become a key strategy to address this issue as network technology is applied to the field of education.

Outliers refer to individual values in a sample, and their values obviously deviate from other values of this group of data. The treatment of outliers should be specifically analyzed according to different situations. We cannot simply reject the outliers directly, which may lead to the loss of useful information or inaccurate results. Therefore, for the small sample dataset, firstly, the outliers are judged, and then the outliers are corrected according to the characteristic analysis deviation and the dispersion of the measured data. After the corrected data is added to the normal data, the final result is obtained.

In statistics, the deviation based on the average value refers to the difference between the average value of all scores of a certain assessed person and the standard value. The deviation based on the correlation deviation means that the standard value is not needed, and the average value of the difference between the evaluation scores of each participating user and other users is calculated as the deviation value. The formula is

(1) $$\begin{array}{c} d_{i}=\frac{1}{n-1}\overset{n}{\underset{i\neq j}{\sum }}\left(A_{i}-A_{j}\right). \end{array}$$

The deviation based on the relative absolute deviation also does not need the standard value, and the average value of the absolute value of the difference between the evaluation scores of each participating user and other users is calculated as the deviation value. The formula is

(2) $$\begin{array}{c} d_{i}=\frac{1}{n-1}\left|\overset{n}{\underset{i\neq j}{\sum }}\left(A_{i}-A_{j}\right)\right|. \end{array}$$

The smaller the number of datasets in small sample data, the greater the influence of outliers on the final result. Mean, variance, standard deviation, etc., are difficult to avoid the influence of gross errors.

The PSO (particle swarm optimization) algorithm adopts the concepts of “colony” and “evolution” and operates according to the fitness of individuals. The structure of the global optimal domain is similar to a fully connected social network, in which each individual can compare with the performance of all other individuals except himself. If an individual finds the optimal solution, all other individuals can be attracted to the optimal solution. Adjust the current particle position and speed according to the following formula:

(3) $$\begin{array}{c} v_{\text{id}}=\omega v_{\text{id}}+c_{1}{\mathrm{rand}}_{1}\left(\right)\left(p_{\text{id}}-x_{\text{id}}\right)+c_{2}{\mathrm{rand}}_{2}\left(\right)\left(p_{\text{gd}}-x_{\text{id}}\right), \end{array}$$

(4) $$\begin{array}{c} x_{\text{id}}\left(t+1\right)=x_{\text{id}}\left(t\right)+v_{\text{id}}\left(t+1\right). \end{array}$$

For a tester, the true score is a constant; *A* is the observation part of multiple measurements, which will fluctuate on the true score *A* when the measurement is realized. Repeat the measurement with parallel tests many times, and the final average score tends to be the true score, namely,

(5) $$\begin{array}{c} \varepsilon \left(A\right)=T. \end{array}$$

In the test paper, there are usually subjective questions and objective questions, so the difficulty of the test questions needs to be calculated separately. The formula of the difficulty coefficient of subjective questions is as follows:

(6) $$\begin{array}{c} q=\frac{x_{i}}{x_{m}}. \end{array}$$

*q* stands for the difficulty coefficient, *x*_*i*_ stands for the average score of the *I*-question test, and *x*_*m*_ stands for the total score of the question.

When the average score of a topic in the test paper is higher, it means that the difficulty coefficient of this topic is smaller. On the contrary, when the average score of a small question is low, the difficulty coefficient of this question is high.

C5.0 is one of the decision tree algorithms, which can generate a multibranch decision tree, and its target variable is the classification variable. Let *A* be taken as the sample set, the objective variable *M* has *s* classifications, *P*(*W*_*i*_, *A*) represents the number of samples belonging to class *W*_*i*_ in *A*, and |*A*| is the number of samples in the sample set *A*; then, the information entropy definition of *A* is

(7) $$\begin{array}{c} I\left(A\right)=-\overset{s}{\underset{i=1}{\sum }}\left(\frac{P\left(M_{i},A\right)}{\left|A\right|}\right)*\log_{2}\left(\frac{P\left(M_{i},A\right)}{\left|A\right|}\right). \end{array}$$

The dimensionless index data is used to standardize the calculation of the evaluation index attribute value. Comprehensive evaluation frequently consists of a significant number of interconnected, mutually restraining, and influential evaluation indicators, all of which have unique aspects. The secret to building a BPNN (BP neural network) is to carefully choose the number of input layers, hidden layers, and output layers, as well as the number of neurons in each. The sigmoid activation function is utilized by the BPNN's buried layer. The sigmoid activation function is expressed mathematically as follows:

(8) $$\begin{array}{c} f\left(x\right)=\frac{1}{1+e^{-x}}. \end{array}$$

The excitation function of the output layer is a pure linear function. The learning rate is an important factor to be considered when establishing the model. In the gradient descent algorithm adopted by BPNN, if the learning rate is too small, the convergence rate will be very slow; if it is too large, the iterative solution will be violently oscillated [21].

The structure of BPNN for calculating the teacher performance evaluation index is shown in Figure 2.

A trained BP network model is able to obtain the evaluation index for the object to be evaluated in accordance with the attribute values of each index; replicate the expertise, knowledge, and subjective assessment of experts and their propensity to emphasize the importance of the index; realize an effective combination of qualitative and quantitative indicators; and ensure the objectivity and consistency of the evaluation. In Figure 3, the algorithm flow for ranking evaluation based on BPNN is displayed.

The evaluation index can be divided into two parts: one is the quantitative index, which can give the score directly according to the scoring standard, and the other is the qualitative index, mainly the teaching quality score. After scoring the qualitative indicators of the *d*th teacher, the expert opinions of each indicator should be collected by the arithmetic average method. Namely,

(9) $$\begin{array}{c} q_{r}=\overset{T}{\underset{s=1}{\sum }}\frac{V_{rs}}{T}, \end{array}$$

where *q*_*r*_ is the expert score of the *d* teacher's *r* index, and *r* is the serial number of the evaluation index.

*V*_*rs*_ is the score of the *r* index of the *d* teacher given by the *s*th expert, *s* is the serial number of the expert, and *r* is an index number; *T* is the effective number of the expert questionnaire.

The purpose of abnormal score correction in the performance evaluation system is to weaken the influence of abnormal scores on the score results. Because the department evaluation is a small sample data, deleting the abnormal value directly will lead to insufficient data. The purpose of correcting the outliers is to make the outliers return to the normal range by calculating the deviation and dispersion so as to reduce the influence on the final result. The final correction formula is

(10) $$\begin{array}{c} A_{\text{new}}=\left\{\begin{array}{c} A_{i}-d_{i}\times Z\;\left(A_{i}>Me\right),\\ \begin{array}{cc} A_{i}+d_{i}\times Z & \left(A_{i}<Me\right). \end{array} \end{array}\right. \end{array}$$

*A*_new_ is the revised evaluation score. *A*_*i*_ is the original score, *d*_*i*_ is the deviation, and *Z* is the dispersion.

## 4. Experiment and Results

The research object of this study selects 300 preschool teachers from 10 urban kindergartens as research samples. In order to ensure that the scales used in this study can accurately measure related variables, this study adopts domestic and foreign mature scales. The researcher invited 10 preschool teachers to conduct in-depth interviews, and they answered them. Based on the preschool teachers' own understanding and feelings of the initial questionnaire items, the researcher summarized their opinions and made corresponding modifications, fine-tuning the problematic and flawed items in the initial questionnaire. Except for demographic variables, the other major variables are scored by the 5-point Likert method, with 1 expressing great disagreement and 5 expressing great agreement. The higher the reliability value, the smaller the error between all the scores of the assessed object. Usually, the reliability value is less than 0.7, which means that the reliability of data is low. When it is close to 0.9, the reliability of the data is high. The reliability analysis of the original data in the library is shown in Figure 4. After the “perfunctory” data and “biased” data are processed, the reliability of the data in the database is analyzed again, as shown in Figure 5.

The reliability after deleting outliers is concentrated in the range of 0.8 to 1, and it can be considered that the outlier processing algorithm is effective. In this paper, descriptive statistics are made on the topics, which mainly include information such as mean, standard deviation, skewness, and kurtosis, so as to judge the basic level of the topics in the scale and the distribution of data presentation.  Table 1 shows the descriptive statistical results of PI.

It can be seen that the PI level of preschool teachers is generally high. Among the four dimensions of PI, the score of occupational behavior tendency is the highest, with an average of more than 4 points, and there is no obvious difference in the average among the dimensions. It shows that teachers are more appreciative of their professional tendencies. On the overall dimension of PI, the standard deviation reached 0.8745, which is the largest value, indicating that in the sense of PI, the subjects had the biggest difference in their views on the dimension of professional belonging. This study investigates the differences of preschool teachers' WE and educational background, age, teaching experience, and marital status, taking educational background, age, teaching experience, and marriage as independent variables and preschool teachers' WE as dependent variables to carry out a one-way ANOVA test. See Table 2 for details.

The results show that marital status (*F* = 0.36, *P* = 0.74) has no significant effect on the primary effect of preschool teachers' WE. Education (*F* = 3.91, *P* = 0.01), age (*F* = 3.14, *P* = 0.01), and teaching experience (*F* = 3.17, *P* = 0.03) have significant main effects on preschool teachers' WE. There is no significant difference in WE scores of preschool teachers between the age group under 25 and the age group between 25 and 35. In terms of teaching age, the scores of preschool teachers with more than five years of teaching age are significantly higher than those of preschool teachers with one year of teaching age, one to three years of teaching age, and three to five years of teaching age. One-way ANOVA shows that there are significant differences in the teaching years of kindergarten teachers' PT (*F* = 3.68, *P* < 0.01), and the results are shown in Table 3.

Generally speaking, with the increase in teaching years, the PT level of preschool teachers also improves. First-time kindergarten teachers scored the lowest on PT, reaching the peak after 16-23 years of teaching experience and then decreasing. The PT of kindergarten teachers in the early career is the lowest, and it reaches the highest in the middle career, and kindergarten teachers in the middle career have more PT than kindergarten teachers in the early career. As shown in Table 4, Pearson's correlation coefficient analysis is carried out with SE and its two dimensions and PT and its three dimensions as variables. The results show that there are significant positive correlations among all factors; that is, the higher the SE level of preschool teachers, the higher their PT level.

There is a significant positive correlation between PI and SE of kindergarten teachers, and SE has a significant positive correlation with WE of kindergarten teachers. It is speculated that SE of kindergarten teachers may play an intermediary role in the relationship between PT and WE. See Table 5 for details.

It can be judged that teachers' SE plays an incomplete intermediary role between PT and WE, with the value of the intermediary effect being 0.041, accounting for 15.7% of the total effect (0.6559). According to the bootstrap results, the 95% confidence interval is [0.1355,0.2186], which does not contain 0, and the mediation effect is significant. After the above neural network training, the weights and thresholds have been determined, and after 20 input values are given, the evaluation results of the neural network can be obtained. The last four groups of data are used for testing, and the evaluation target obtained after the result is subjected to inverse normalization processing is compared with the actual evaluation target so that the testing error of the network can be obtained, which is shown in Figure 6.

The test results can be seen to be quite near to the actual data, demonstrating that the model is capable of precisely determining the teaching effect for each assessment measure. The error signal will automatically adjust, and the phenomena of training approaching the saturation area will be avoided if the derivative of the excitation function is changed. This will speed up the algorithm's convergence and enhance its capacity for global convergence. This paper proposes an enhanced BP technique for adaptive error signals. A number between [0, 1] is randomly chosen as the initial weight in the BP network, and the original value is sampled with a step size of 0.05. Figures 7 and 8 display the simulation results following 100 experiments.

From the above simulation results, it can be seen that the average iteration steps of the improved algorithm are obviously less than those of the standard BP algorithm, which indicates that the improved algorithm converges faster, the function approximation effect of the improved algorithm is better, and the network training is more stable.

## 5. Conclusion

Children's speech should be positive, pay attention to internal attribution, be as specific as possible, and be equipped with appropriate tone and manner. Because a teacher's speech affects the teacher-child relationship, a good teacher-child relationship can meet the learning and emotional needs of children. The results of this study show that the standard deviation of PI is 0.8745, which is the largest value, indicating that in the sense of PI, the subjects have the biggest difference in the sense of professional belonging. Marital status (*F* = 0.36, *P* = 0.74) has no significant effect on the primary effect of preschool teachers' WE. Education (*F* = 3.91, *P* = 0.01), age (*F* = 3.14, *P* = 0.01), and teaching experience (*F* = 3.17, *P* = 0.03) have significant main effects on preschool teachers' WE. SE plays an incomplete intermediary role between PT and WE, with the value of the intermediary effect being 0.041, accounting for 15.7% of the total effect (0.6559).

## Figures and Tables

**Figure 1:** Research model design.

**Figure 2:** BPNN structure for calculating the teacher performance evaluation index.

**Figure 3:** Algorithm flow of BPNN ranking evaluation.

**Figure 4:** Reliability analysis of original data.

**Figure 5:** Reliability analysis of postprocessing data.

**Figure 6:** Error test result.

**Figure 7:** Function approximation effect of the standard BP algorithm.

**Figure 8:** Function approximation effect of the improved BP algorithm.

**Table 1:** PI descriptive statistics.

Dimension	Minimum	Maximum	*M*	SD
Role values	1.487	6	3.3127	0.7092
Professional behavior tendency	1.184	6	3.0961	0.8679
Professional values	1.2145	6	3.5695	0.667
Professional sense of belonging	1.2774	5.53	3.6542	0.7007
PI population	1.0961	6	3.7445	0.8745

**Table 2:** Mean and standard deviation of preschool teachers' WE.

Project		*M*	SD	*F*	
Academic degree	Technical secondary school	3.8958	0.4782	3.688^∗^	^∗^ *P* < 0.05
	Universities and colleges	3.8132	0.4637		
	Bachelor's degree or above	3.9145	0.4447		
Age	Under 25 years old	4.0954	0.4662	3.55^∗^	
	25 to 35 years old	3.5785	0.4784		
	Over 35 years old	4.3678	0.462		
Length of teaching	Less than 1 year	4.1395	0.4343	3.17^∗^	
	1 to 3 years	4.3017	0.494		
	3 to 5 years	4.3205	0.4936		
	More than 5 years	3.755	0.4108		

**Table 3:** The difference test of kindergarten teachers' PT in teaching age.

		*M*	SD	*F*	
Length of teaching	Less than 1 year	4.3527	0.4827	3.62^∗∗^	^∗∗^ *P* < 0.01
	1 to 3 years	4.6326	0.491		
	3 to 5 years	4.4419	0.4335		
	More than 5 years	4.4179	0.4848		

**Table 4:** Correlation matrix of SE and PT.

Dimension	General SE	Individual SE	SE
Overcome difficulties	0.2184	0.696	0.5861
Coping with stress	0.2423	0.6224	0.5805
Rejuvenation	0.2695	0.6101	0.5804
PT	0.2384	0.6284	0.5147

**Table 5:** Bootstrap analysis results of the intermediary effect significance test.

Effect type	Effect value	Boot SE	Bootstrap (95% CI)		Relative effect ratio (%)
			Lower limit	Upper limit	
Total effect	0.6559	0.0716	0.3603	0.4482	100
Direct effect	0.3204	0.0349	0.2142	0.2296	84.3
Indirect effect	0.041	0.0416	0.1355	0.2186	15.7

## Data Availability

The data used to support the findings of this study are available from the corresponding author upon request.
